# 5-aminosalicylic acid improves lipid profile in mice fed a high-fat cholesterol diet through its dual effects on intestinal PPARγ and PPARα

**DOI:** 10.1371/journal.pone.0191485

**Published:** 2018-01-19

**Authors:** Zheng Wang, Debby Koonen, Marten Hofker, Zhijun Bao

**Affiliations:** 1 Department of Geriatrics and Gastroenterology, Huadong Hospital, Shanghai Medical College, Fudan University, Shanghai Key Laboratory of Clinical Geriatric Medicine, Shanghai, P.R. China; 2 Department of Pediatrics, Section Molecular Genetics, University Medical Center Groningen, University of Groningen, Groningen, the Netherlands; INRA, FRANCE

## Abstract

Obesity is associated with a series of metabolic complications, including dyslipidemia and insulin resistance (IR) that lack effective therapies. In recent years, intestinal inflammation has been suggested to contribute to obesity related metabolic syndrome and targeting gut inflammation with 5-ASA improves diet induced IR, however, its role in dyslipidemia is unknown and has never been explored. In the present study, we reported for the first time that administration of 5-ASA for 12 weeks significantly improved lipid profile by repressing plasma triglycerides and free cholesterol levels in mice fed high-fat cholesterol diet (HFC). In addition, liver lipids were significantly reduced by 5-ASA treatment in HFC-fed mice. Mechanistically, anti-inflammatory genes peroxisome proliferator-activated receptor-γ (Pparγ) and M2 marker, such as Mrc1 and Ym1, were remarkably upregulated, while pro-inflammation gene monocyte chemoattractant protein-1 (Mcp-1) were downregulated in small intestine of mice treated by 5-ASA. Further, 5-ASA improved gastrointestinal barrier by increasing the expression of the tight junction marker ZO-1. 5-ASA also enhanced cholesterol translocation by elevating genes expression of Npc1l1 and Abcg5/8. Moreover, mice fed HFC 5-ASA expressed increased Pparα in small intestinal and its target genes function in lipid oxidation and hydrolysis were remarkable elevated. Taken together, we reported a novel role of 5-ASA which may serve as a therapy target intestinal inflammation induced dyslipidemia.

## Introduction

Obesity is emerging as a global public health problem and is associated with a series of metabolic complications, including dyslipidemia and insulin resistance (IR) whereas the mechanism is not fully understood. Numerous studies have shown that activation of intestinal inflammation is strongly associated with early on-set obesity and plays a causal role in the development of obesity related metabolic syndrome [1, 2]. These studies suggest that strategies, which reduce intestinal inflammation, maybe useful for therapy of IR, dyslipidemia and cardiovascular disease [3].

5-aminosalicylic acid (5-ASA, also known as mesalamine) is a salicylic acid derivative with anti-inflammatory properties. Since its introduction, 5-ASA has proven effective in both the maintenance and treatment of Crohn’s disease and ulcerative colitis, two principal forms of chronic inflammatory bowel disease (IBD). After oral or rectal administration, 5-ASA is absorbed by intestinal epithelial cells and acts locally in the gut while systemic dosages remain low [4]. Although the clinical safety and efficacy of 5-ASA has been well known, the related mechanism of its action has not been fully elucidated[5–9]. A number of anti-inflammatory actions of 5-ASA have been proposed, including inhibition of the activity of nuclear factor-kappa B (NF-κB) by modulating RelA/p65 phosphorylation [10], and reduction of the biosynthesis of prostaglandins and leukotrienes [11, 12]. Moreover, 5-ASA shares many of the pharmacological properties of non-steroidal anti-inflammatory drugs (NSAIDs) such as aspirin. Recently, 5-ASA was shown to exert its anti-inflammatory effects through the activation of nuclear receptor peroxisome proliferator-activated receptor-γ (PPARγ) [7]. Expressed at high levels in the intestinal epithelium, PPARγ plays an important role in the maintenance of mucosal integrity and in the regulation of epithelial inflammatory response [13]. In addition, PPARγ activation leads to a cascade of events that controls the expression of a large number of regulatory genes in lipid metabolism as well as insulin sensitization [14] and in recent years, PPARγ has emerged as link between lipids, metabolic diseases and innate immunity [15].

Recently, 5-ASA was shown to reverse bowel inflammation and improve systemic metabolic parameters and insulin resistance during high-fat feeding in mice [16]. In this study, histological evidence indicated a reduction in liver steatosis in 5-ASA-treated mice [16], however, plasma and hepatic lipid levels were not quantitatively measured. In addition, 5-ASA is absorbed by intestinal epithelial cells in the proximal gastrointestinal tract [17], where the enterocytes are the primary cells involved in dietary lipid digestion and absorption [18]. These observations raise the possibility of 5-ASA to act as a lipid regulatory agent, however, a therapeutic role for 5-ASA in the management of dyslipidemia and the potential mechanism has never been explored.

Here, we hypothesized that 5-ASA might have lipid-lowering effects through its effect on intestine. Our results demonstrate that oral 5-ASA administration improve lipid profile especially when mice were fed a high-fat, cholesterol-rich diet. 5-ASA treatment brought down inflammation related genes expression, led to a shift from M1 to M2 macrophages and activated PPARα related fatty lipid oxidation in small intestine. Based on these findings, we proposed that gut inflammation may play an important role in intestinal lipid metabolism and 5-ASA may thus serve as a novel modulator to ameliorate dyslipidemia in metabolic disease.

## Materials and methods

### Mice and treatment

This study was carried out in strict accordance with the recommendations in the Guide for the Care and Use of Laboratory Animals of the Netherlands. The protocol was approved by the Ethical Committee for Animal Experiments of the University of Groningen and the Institutional Animal Care and Use Committee of Huadong hospital affiliated to Fudan University (Permit Number: 15246.2) and the methods were carried out in accordance with the approved guidelines. All surgery was performed under isoflurane anesthesia, and all efforts were made to minimize suffering. Experiments were carried out on male C57BL/6J mice purchased from Charles River (France). The animals were acclimatized to laboratory conditions (23°C, 12h/12h light/dark) for one week prior to experimentation. Mice were housed separately in Individual Ventilated Cages with ad libitum access to food and water. Mice were randomized in 4 groups of 10 mice each. Mice were fed either low-fat diet (LFD; 10% kcal fat, Research Diets), LFD 5-ASA, high-fat diet supplemented with 0.25% cholesterol (HFC; 60% kcal fat, Research Diets) or HFC 5-ASA starting at 10–12 weeks of age. Mice were kept on these diets for 12 weeks. Animals were sacrificed by cardiac puncture under isoflurane anesthesia. Anesthesia was induced with 4% isoflurane (Isofluran CPR, CP-Pharma Handelsgesellschaft mbH, Burgdorf, Germany) in 100% oxygen in an anesthetic chamber (with sliding cover, Evonik Plexiglas, 240 × 140 × 120 mm), which was not prefilled in order to prevent distress.Liver tissue was collected and snap-frozen in liquid nitrogen or fixed in formalin. Intestines were flushed and snap-frozen in liquid nitrogen.

### Compounds and metabolic studies

5-ASA powder (Sigma-Aldrich) was mixed into the LFD and HFC diets at 1,500 mg/kg/day. All diets were prepared fresh weekly to ensure a consistent 5-ASA dose intake of 1,500 mg/kg/day throughout the 12-week dietary intervention study. Body weight and food intake was measured weekly. After 11 weeks on LFD or HFC, mice were fasted for 6 hours to measure the blood glucose level using OneTouch Select plus glucose meter (LifeScan Benelux, Johnson & Johnson Medical BV). In addition, blood samples were collected in EDTA-coated tubes for determination of insulin levels. Samples were spun at 3000rpm for 10 min at 4°C and insulin concentrations were measured in plasma using a commercially available ELISA kit (Alpco Diagnositics, Salem, NH). One day prior to sacrifice body composition was analysed using a Minispec Whole Body Composition Analyser (Bruker).

### Quantification of plasma and liver lipids

Plasma triglycerides, total cholesterol and free cholesterol were determined at times of sacrifice using commercially available kits (Triglycerides and total cholesterol: Roche; free cholesterol: FS DiaSys, Holzheim, Germany). To measure hepatic lipid content, lipids were extracted from crushed liver samples using Bligh and Dyer’s method [19]. Hepatic triglyceride and cholesterol levels were measured using kits that are commercially available (Triglycerides and total cholesterol: Roche; free cholesterol: FS DiaSys).

### Histology

For microscopic examination, liver tissues were fixed in 4% (w/v) phosphate-buffered formalin, embedded in paraffin, sectioned at 4μm and stained with hematoxylin and eosin (H&E). Representative photomicrographs were captured at 100× magnification using the software incorporated in the microscope (Leica DM 3000).

### Quantitative real-time PCR (qPCR)

RNA was isolated using Qiazol reagent, according to the manufacturer’s instructions (Roche). cDNA was synthesized using the Transcriptor Universal cDNA Master kit from Roche, according to their instructions (Roche, Mannheim, Germany). We performed quantitative real-time PCR with a 7900HT PCR system (Applied Biosystems) using SYBR Green Master Mix reagent (Roche). Each sample was run in triplicate and normalized to PPIA as housekeeping gene. We calculated relative fold changes in gene expression normalized to PPIA by the ΔΔCT method using the equation 2^-ΔΔCT^. The results are shown as fold changes compared to the HFC group. Primer sequences are listed in S1 Table.

### Statistical analysis

The data were presented as mean ± SEM. Comparisons between groups were performed using unpaired Student’s two-tailed t tests in GraphPad Prism 5. P < 0.05 was considered statistically significant.

## Results

### Body weight, food intake and glucose levels were not affected by 5-ASA in LFD-fed mice

To examine the effects of 5-ASA on weight gain and body composition, we fed C57BL/6J mice with either low-fat diet (LFD) or LFD incorporated with 5-ASA for 12 weeks. By the end of week 12, mice from these two groups did not show differences in body weight (Fig 1A) and fat or lean mass were similar (Fig 1B). Furthermore, there was no effect of 5-ASA on food intake (Fig 1C) or fasting glucose (Fig 1D). However, mice receiving 5-ASA showed a trend towards lower plasma triglycerides (0.91±0.12 vs. 0.59±0.10, P = 0.052, Fig 1E), whereas no effect was seen on the plasma levels of free (Fig 1F) and total cholesterol (Fig 1G).

**Fig 1:** 5-ASA treatment does not affect the metabolic parameters in mice fed LFD. (A) Body weights of LFD and LFD 5-ASA-fed C57BL/6J mice over time, starting at 10–12 weeks of age. (B) Fat or lean mass, expressed as percentage of body weight, were analyzed after 12 weeks of LFD or LFD 5-ASA. (C) Food intake of mice fed LFD and LFD 5-ASA at the first week and week 11. (D) Fasting glucose of 11-week LFD or LFD 5-ASA-fed mice. (E-G) Plasma triglycerides, free cholesterol and total cholesterol were quantitatively analyzed in mice fed 12 weeks of LFD or LFD 5-ASA. Data are presented as means ± SEM, n = 9–10 mice.

### 5-ASA treatment improves plasma lipid levels in HFC-fed mice

To assess whether 5-ASA may improve plasma lipid levels in the setting of diet-induced obesity (DIO), we challenged C57BL/6J mice with either a HFC diet or HFC incorporated with 5-ASA for 12 weeks. Consistent with 5-ASA treatment in mice fed LFD, 5-ASA did not change body weight (Fig 2A), fat or lean mass (Fig 2B) or food intake (Fig 2C) in mice fed a HFC diet. In contrast to the recently reported beneficial metabolic effects of 5-ASA on insulin resistance in high-fat diet (HFD)-fed mice[16], we did not observe improvements in fasting glucose (Fig 2D) or fasting insulin (Fig 2E) in HFC-fed mice receiving 5-ASA. However, plasma triglycerides were significantly reduced in 5-ASA treated HFC-fed mice (0.59±0.04 vs. 0.48±0.02, Fig 2F). Furthermore, mice receiving 5-ASA showed a significant reduction in free cholesterol levels (1.29±0.03 vs. 1.12±0.05, Fig 2G), whereas total cholesterol level was unchanged (Fig 2H). These results suggest that 5-ASA may act as a lipid-lowering agent in dyslipidemic settings.

**Fig 2:** 5-ASA treatment attenuates plasma lipid levels in HFC-fed mice. (A) Body weights of HFC and HFC 5-ASA-fed C57BL/6J mice over time, starting at 10–12 weeks of age. (B) Fat or lean mass to body weight ratio were assessed after 12 weeks of HFC or HFC 5-ASA. (C) Food intake of mice fed HFC and HFC 5-ASA at the first week and week 11. (D-E) Fasting glucose and fasting insulin of mice after 11 weeks of HFC or HFC 5-ASA. (F-H) Plasma triglycerides, free cholesterol and total cholesterol levels of 12-weeks HFC or HFC 5-ASA-fed mice. Data are presented as means ± SEM, n = 9–10 mice, ^a^P < 0.05 vs. HFC, ^b^P < 0.01 vs. HFC.

### 5-ASA treatment alleviates liver lipid accumulation in mice fed a HFC-diet

Since the liver plays an important role in maintaining lipid homeostasis, we investigated if 5-ASA treatment may also result in reduced lipid accumulation in the liver in mice fed a HFC diet for 12 weeks. Liver weight was not different between 5-ASA treated and non-treated HFC-fed mice (Fig 3A) and visual inspection of H&E stained liver slides did not show obvious signs of 5-ASA treatment on lipid accumulation in HFC-fed mice (Fig 3B). However, following lipid extraction of liver tissue we observed a significant reduction in triglycerides (76.43±8.01 vs. 55.27±3.43, Fig 3C), but not total (Fig 3D) and free cholesterol (Fig 3E) in the livers of 5-ASA treated versus non-treated HFC-fed mice.

**Fig 3:** 5-ASA treatment alleviates hepatic lipid accumulation during HFC feeding. (A) Liver weights were measured on sacrifice day after 12 weeks of HFC or HFC 5-ASA. (B) Histology of liver after 12 weeks of either HFC or HFC 5-ASA diet (H&E stain; 100×). (C-E) Hepatic triglycerides, total cholesterol and free cholesterol levels of HFC or HFC 5-ASA-fed mice. Data are presented as means ± SEM, n = 9–10 mice, ^a^P < 0.05 vs. HFC.

### Effects of 5-ASA intervention on inflammation and tight junction of the small intestine

To determine the anti-inflammatory actions of 5-ASA, firstly we conducted qPCR in small intestine and found the mRNA expression of Pparγ in HFC 5-ASA group was 1.79 times higher than HFC group (Fig 4A). Although genes expression of interleukin 6 (Il6), a pro-inflammatory macrophage (M1) marker, was not affected, anti-inflammatory macrophage (M2) markers, Mrc1 and Ym1, expressions were significantly increased (Fig 4A) and inflammatory genes monocyte chemoattractant protein-1 (Mcp-1) was brought down to 0.66 times in the HFC 5-ASA group compared with HFC group (Fig 4A). In addition, HFC 5-ASA group displayed higher level of expression of Zo-1 (Fig 4B), a key tight junction marker, suggesting that 5-ASA down regulated gut inflammation and improved intestinal barrier.

**Fig 4:** Effects of 5-ASA intervention on inflammation and tight junction of the small intestine. (A) qPCR analysis of small intestinal lysates for gene expression of PPARγ, IL-6, Mrc1, Ym1 and MCP1. (B) qPCR analysis of small intestinal lysates for gene expression of ZO-1. Data are presented as means ± SEM, n = 9–10 mice, ^a^P < 0.05 vs. HFC, ^b^P < 0.01 vs. HFC, ^c^P < 0.001 vs. HFC.

### 5-ASA enhanced lipid translocation and fatty acid oxidation in small intestine

Given 5-ASA administration unregulated PPARγ, as expected, we detected a 2.08 times increase of Cd36 mRNA expression in small intestine (Fig 5A). As a downstream target gene of PPARγ, CD36 is known as the mediator in long chain fatty acid (LCFA) uptake, however, other crucial genes function in LCFA uptake, such as Fatp4 and L-fabp, were remain unchanged (Fig 5A). Besides, mRNA expression of intestinal cholesterol transporters Abcg5, Abcg8 and Npc1l1 were all increased in mice fed HFC 5-ASA relative to mice fed HFC (Fig 5B), suggesting that 5-ASA may enhanced both cholesterol absorption and excretion.

**Fig 5:** Effects of 5-ASA intervention on lipid translocation in small intestine. (A) qPCR analysis of small intestinal lysates for gene expression of CD36, FATP4 and L-FABP. (B) qPCR analysis of small intestinal lysates for gene expression of ABCG5, ABCG8 and NPC1L1. Data are presented as means ± SEM, n = 9–10 mice, ^a^P < 0.05 vs. HFC.

It is known that activation of the PPARs family leads to multiple beneficial outcomes. PPARα agonist is reported associated with improvement in lipid profiles, including lowering triglyceride level in diabetes patients. Thus, we hypothesis the lipid lowering effect of 5-ASA is mediated by PPARα. As we expected, mice fed HFC 5-ASA showed a significant higher Pparα gene expression in small intestines when compared to HFC-fed mice (Fig 6A), suggesting that 5-ASA regulated lipid metabolism in multiple metabolic pathways and prompting us to further explore the expression of PPARα target genes involved in lipid oxidation in small intestine. Indeed, HFC-fed mice treated with 5-ASA exhibited dramatically increased expression of hormone-sensitive lipase (Hsl), which play roles in lipolysis and energy metabolism (Fig 6B). Several mitochondrial fatty acid oxidation enzyme genes (Aox, Aco, Ctp1α, Mcad) expression were all increased as well in mice fed HFC 5-ASA group compared to mice fed HFC diet (Fig 6C).

**Fig 6:** Effects of 5-ASA intervention on fatty acid oxidation in small intestine. (A) qPCR analysis of small intestinal lysates for gene expression of PPARα. (B) qPCR analysis of small intestinal lysates for gene expression of Desnutrin and HSL. (C) qPCR analysis of small intestinal lysates for gene expression of AOX, ACO, CPT1α and MCAD. Data are presented as means ± SEM, n = 9–10 mice, ^a^P < 0.05 vs. HFC, ^b^P < 0.01 vs. HFC.

## Discussion

Current findings support views that anti-inflammation may help to prevent, reverse and alleviated associated complications [20, 21]. Drugs targeting inflammatory pathways are in trials and have shown some efficacy in rodents and clinical studies. For example, TNFα blocking agents and IL-1**β** have marked effects to improve insulin sensitivity and lower blood glucose levels in rodents[3, 22]. Although promising, the observed metabolic effects remain rather modest in most clinical trials and along with potential serious side effects[23–25]. Intestinal inflammation is emerging revealed as an early event in obesity and type 2 diabetes mellitus (T2DM), and mediates the development of related metabolic complications, such as insulin resistance, dyslipidemia and cardiovascular diseases [3, 26]. Evidence suggested that intestinal inflammation is an early consequence of HF diet that may contribute to obesity related complications[16, 26]. Interventions which limit intestinal inflammation induced by HF diet may protect against obesity and insulin resistance[16, 26] The key new findings of this study are that, gut specific anti-inflammatory agent 5-ASA has a lipid lowering effect in mice fed HFC diet, including reduction of plasma triglyceride as well as free cholesterol concentrations and alleviation of hepatic lipid accumulation. These findings revealed the role of intestinal inflammation in the development of diet-induced dyslipidima. We also report for the first time that the lipid-lowering effect of 5-ASA is associated with enhanced PPARα related fatty acid oxidation in the small intestine.

5-ASA is widely used in the treatment of IBD and is among the oldest anti-inflammatory agents in use today. After oral or rectal administration, 5-ASA acts locally in the colon and is absorbed by colonic epithelial cells[27–29]. Although the exact mechanisms of action of 5-ASA are not completely elucidated, recent studies have revealed that the basic mechanism of action of 5-ASA is relying on increased expression of PPARγ [7]. As a prototype of a new class of PPARγ agonists, 5-ASA increased PPARγ expression, promoted its translocation from the cytoplasm to the nucleus, and induced a modification of its conformation permitting the recruitment of co-activators and the activation of a peroxisome-proliferator response element-driven gene[7, 30]. PPARs are members of the nuclear receptor superfamily and expressed at high levels in the intestine epithelium[31]. In addition to its efficacy as an anti-inflammatory target, PPARγ is believed to act as a main lipid sensor controlling the expression of genes that function in lipid and carbohydrate metabolism [15], resulting in increased expression of lipoprotein lipase (LPL) and decreased expression of apolipoprotein (apo) C-III, both key-players in plasma triglyceride metabolism[32]. Full PPARγ agonists, such as thiazolidinediones, are a novel class of anti-diabetic drugs and also exert lipid lowering function, however, these agents shall thus avoid adverse effects, such as body weight gain[33, 34]. Our data showed that 5-ASA upregulated PPARγ, lowered triglycerides level in mice fed HFC (Fig 3B and 3C), but did not affect body weight (Figs 1A and 2A). We infer 5-ASA may act as a novel class of non-thiazolidinedione partial PPARγ ligands, which is expected to benefit from lipid profile without adverse effects mentioned above by preferential recruitment of PPARγ-coactivator-1α (PGC1α) to the receptor, a feature shared with other selective PPARγ modulators, to prevent triglyceride accumulation[35]. Collectively, that information and our data suggest the regulatory potential of 5-ASA in lipid metabolism.

Our data showed the anti-inflammatory effect of 5-ASA by increasing PPARγ and reducing Mcp-1 genes expression in small intestine (Fig 4A), however, M1 marker, Il-6 were not significantly altered. Surprisingly, we noticed a remarkable higher expression of M2 marker, such as Mrc1 and Ym1, suggesting 5-ASA may contribute to a shift from pro-inflammation to anti-inflammation macrophages. It is well established that M1 activity result in tissue damage while M2 activity promotes tissue repair [36], and in our study, we indeed found that the tight junction marker Zo-1 expression was more abundant after 5-ASA treatment. Moreover, previous study reported PPARγ played a critical role in the maintenance of intestinal mucosal integrity [13, 31]. Taken together, our data indicate 5-ASA reduced intestinal inflammation and strengthened the gut barrier, which are associated with reduced gut permeability and endotoxemia, and ultimately contribute to the improved metabolic parameters [16].

Our findings (anti-gut inflammatory agent showed lipid lowering effect) are in line with a preclinical analysis in which they demonstrated the long-term administration of NSAIDs, the widely used systemic anti-inflammatory therapies, was useful for preventing steatohepatitis and atherosclerosis in mice fed a HFD [37] Moreover, high dose Aspirin, one of the typical NSAIDs, also known as acetylsalicylic acid, impressively reduces total cholesterol levels by 50% and significantly reduce hepaticsteatosis [37]. T2DM patients taking Aspirin also benefit from decreased serum total cholesterol (~15%) and triglycerides (~50%) [38]. Although the lipid lowering effect of 5-ASA is fairly mild (19% reduction in plasma triglyceride levels), the primary advantage of 5-ASA is it acts locally in the gut and well tolerated even at a high dose, which is different from the systemic anti-inflammatory therapies such as Aspirin, carrying potential serious side effects.

Another novel finding in our study is ABCG5/8 and NPC1L1 were upregulated in small intestine after 5-ASA treatment (Fig 5B), to our knowledge, which is never been reported before. The ABCG5/ABCG8 heterodimer promotes cholesterol removal from the body and intestinal ABCG5/ABCG8 responsible for extrahepatic cholesterol efflux [39]. On the contrary, NPC1L1 is a sterol transporter that mediates intestinal cholesterol absorption [40]. Surprisely, 5-ASA seems enhance both cholesterol absorption and excretion, however, we infer the increased expression of NPC1L1 maybe a compensatory consequence of enhanced cholesterol efflux and it also indicated that the function of small intestine is recovered together with the strengthened wall of gut. Further studies are needed to understand the mechanism and to clarify the net effect of absorption and excretion.

In addition, we observed a significant increase expression of PPARα gene as well as its target genes function in lipolysis and fatty acid β-oxidation in small intestine of 5-ASA treated mice (Fig 6A–6C). PPARα is expressed at high levels in both human and murine small intestine, especially in villus cells of proximal small intestine, and has emerged as target for anti-inflammatory activity and lipid-modifying properties[15, 41–44]. Disruption of the PPARα gene in mice revealed its role in fatty acid oxidation, fatty acid uptake and lipoprotein assembly and transport[45]. Fibrates, agonists of PPARα, has been proved fairly successful in clinical at treating dyslipidemia by stimulating fatty acid oxidation in the liver[46] and in reducing the risk of major cardiovascular events[47]. Although there is hardly any literature notice the effect of 5-ASA on PPARα, it seems reasonable to observed the up-regulation gene expression of PPARα in HFC 5-ASA treated groups (Fig 6A). Since members of PPARs family not only share certain conformations but also their regulation effects on lipids metabolism and inflammation [15]. However, further studies are urgently needed to explore the specific interaction between them. For mice receiving low-fat diet (LFD), we did not observed differences in plasma lipid profile or hepatic lipid level (Fig 1E, 1F and 1G). In line with this, there is no difference in PPARγ or PPARα gene expression between LFD and LFD 5-ASA groups. In line with our data, previous study showed that 5-ASA regulated obesity-related insulin resistance in HFD feeding mice, but not affect metabolic parameters in LFD feeding mice[16]. Hence, we infer that the effect of 5-ASA may also dependent on individual metabolic status.

Taken together with the beneficial effects of PPARγ, agonism of both PPARγ and PPARα could potentially benefit T2DM patients with dyslipidemia. Our findings indicate that 5-ASA may control blood lipid levels through a dual PPARγ- and PPARα -mediated effect in the small intestine.

In contrast with previous study, we did not see improvements in fasting glucose and insulin levels following 5-ASA treatment on both LFD conditions and under DIO settings (Figs 1D, 2D and 2E). This contrasted with the study by Luck et al, who reported a beneficial effect of 5-ASA treatment in IR related metabolic parameters[16]. Although we cannot explain this conflicting finding, it may perhaps be related to the younger starting age of the mice in the study by Luck et al. (6 weeks of age vs. 12 weeks), the different composition of the diet (HF vs. HFC) or to more consistent 5-ASA dosing in our study as we prepared the 5-ASA diet fresh every week to correct for body weight gain in the mice. Thus, we recommend that therapies for IR based on anti-gut inflammation should be interpreted with caution.

## Supporting information

S1 Table Primer sequences used for qPCR. (DOCX)
